This article has been retracted.

# Effect of Ruanjian Xiaoying Granules on Hashimoto Rats with Depression of Liver and Deficiency of Spleen and Effect on Intestinal Microflora

**DOI:** 10.1155/2022/8221124

**Published:** 2022-06-28

**Authors:** Tianjiao Dong, Lan Zhang

**Affiliations:** ^1^First Clinical College, Liaoning University of Traditional Chinese Medicine, Shenyang 110847, China; ^2^Endocrinology, Affiliated Hospital of Liaoning University of TCM, Shenyang 110032, China

## Abstract

In order to investigate the effect of Ruanjian Xiaoying Granule, experiments were conducted on the intestinal flora of rats with liver depression and spleen deficiency. 48 SPF grade rats are used as the object, and 12 rats are randomly selected as the normal control group. The Hashimoto rat model of liver depression and spleen deficiency type by drug intervention is constructed by the remaining rats. They are randomly divided into three groups: the model group, the traditional Chinese medicine group, and the Jinshuibao group. The normal group and model group are given 2 ml of distilled water twice a day, and the traditional Chinese medicine group is given the Ruanjian Xiaoying granule group (12.96 g/kg/day) twice a day. The Jinshuibao capsule is dissolved in water and given orally at a dose of 0.45 g/kg/day twice a day. After 12 weeks of intervention, the effect is evaluated, and the levels of serum TGAb, TPOAb, and bacterial diversity are compared. Experimental results show that Ruanjian Xiaoying granules can promote the regulation of flora levels in Hashimoto rats with liver depression and spleen deficiency.

## 1. Introduction

Hashimoto's thyroiditis is a chronic autoimmune disease with its own thyroid tissue as an antigen [1]. There are many kinds of autoimmune thyroid diseases. Hashimoto's thyroiditis is one of them. Hashimoto's thyroiditis patients may have autoantibodies against the thyroid gland, which can induce and cause immune inflammatory damage to the thyroid gland. Common thyroid autoantibodies include antithyroid peroxidase antibody, antithyroglobulin antibody, antithyroid microsomal antibody, etc. The induced autoimmune changes are usually manifested by a large number of lymphocyte infiltration in the thyroid tissue, which will lead to goiter in patients. Some patients are prone to functional abnormalities, mainly hypothyroidism. Epidemiological investigation results show that Hashimoto's thyroiditis has a worldwide prevalence rate of about 2%, and the incidence rate in males is lower than that in females [2]. It is generally believed that the incidence of Hashimoto's thyroiditis is related to genetic, immune, and environmental factors. Like Graves' disease, both of them are specific autoimmune diseases [3, 4]. The early symptoms of Hashimoto's thyroiditis are not obvious. With the prolongation of the disease, it can induce goiter, increase or decrease the incidence, and in severe cases, thyrotoxicosis will increase, affecting the normal life and health of patients. Traditional Chinese medicine believes that Hashimoto's thyroiditis belongs to the category of “gall disease,” and its mechanism is relatively more related to the patient's mood and diet, resulting in liver depression and spleen deficiency, as well as body dysfunction [5]. The Ruanjian Xiaoying granule is a commonly used Chinese medicine granule in clinical practice. Based on Xiaoyao Powder in Taiping Huimin Medicine Bureau Prescription, the effect of soothing the liver and invigorating the spleen can be detected. The Ruanjian Xiaoying granules can reduce the TGAb and TPOAb levels of Hashimoto's thyroiditis by adding and subtracting according to Professor LAN Zhang. Inhibition of TLRs/MyD88/NF-*κ*B signaling can reduce apoptosis in Hashimoto's thyroiditis [6]. Good effects can be obtained in Hashimoto's thyroiditis, but there are few studies on the effect of drugs on the intestinal flora of Hashimoto rats.

The remainder of this paper is organized as follows: Section 2 discusses related work.  Section 3 is the animal data. Our proposed method is followed in Section 4. Experimental data are discussed in Section 5. Finally, the conclusions are presented in Section 6.

## 2. Related Work

The pathogenesis of Hashimoto's thyroiditis is complex and belongs to the category of “gall disease” in Traditional Chinese medicine. Due to the joint action of a variety of factors, it leads to liver depression, spleen deficiency, and body dysfunction. The Ruanjian Xiaoying granule is a Chinese patent medicine commonly used in clinical practice, and the results of previous studies have confirmed that the soft Jian Xiaoying granule based on liver-soothing and spleen-strengthening components can significantly reduce the level of thyroid autoantibodies and achieve good results [7]. Ruanjian Xiaoying granule is mainly composed of Bupleurum, Poria cocos, Atractylodes atractylodes, Angelica, Paeonia alba, seaweed, and kelp. Among prescriptions, Bupleurum has the effect of relieving fever and relieving depression; Tuckahoe has the effect of nourishing water and detumescence, invigorating the spleen and stopping diarrhea, nourishing the heart and calming the mind. Atractylodes macrocephala (ATractylodes macrocephala) has the functions of invigorating the spleen and supplementing qi and regulating gastrointestinal movement. Angelica has the function of invigorating blood circulation, regulating menstruation, and relieving pain; Radix Paeonia has antispasmolysis, antiinflammation, and enhancing immune function. Seaweed can protect the elasticity of blood vessels, reduce cholesterol content, and play an effect on water detumescence. Kelp has the effect of eliminating phlegm and swelling. All drugs played together, can promote thyroid function to return to normal, and can get a good prognosis.

Hashimoto's thyroiditis is a type of autoimmune thyroid disease characterized by slow and inconspicuous progression. Thyroid tissue contains a large number of lymphocytes and lymphatic follicles. Lymphocytes and part of thyroid tissue cells can secrete different cytokines, such as TNF-*α*, IL-2, IL-6, etc., which have strong cytolysis function and have a certain regulation ability on the interaction between thyroid cells and inflammatory cells [8]. In terms of immune factors, with the increase of research on IL-17 in recent years, a new CD4T cell subgroup, namely Th17, has been discovered, which is a T-cell-derived factor and can promote the release of IL-6 and IL-2 and other pro-inflammatory factors [9]. Considering that Hashimoto's thyroiditis induces and participates in the occurrence and development of human autoimmune diseases by secreting the same IL-6 and IL-2 cytokines in lymphocytes and part of thyroid tissue cells as IL-17, it can be inferred that IL-17 is involved in the occurrence and development of Hashimoto's thyroiditis.

Studies have shown that the spacing and thickness of two adjacent microvilli in the intestinal tract of patients with autoimmune thyroiditis are different from those of normal people, suggesting that the intestinal barrier is damaged, which changes the intestinal environment and leads to the occurrence of immune diseases. The intestinal flora can improve or destroy the intestinal mucosal barrier [10]. Also, it can improve or promote the process of immune diseases in the human body [11]. The occurrence of liver depression and spleen deficiency is Hashimoto's a multifactor process, often accompanied by gastrointestinal flora disorder. The flora of the human gastrointestinal tract is more complex and the number is relatively large, which contains both beneficial bacteria and pathogenic bacteria, and can be transformed into each other under specific conditions, thus inducing other diseases. In this study, it was found that firmicutes increased in the model group compared with the normal group at phylum level, while firmicutes decreased after Ruanjian Xiaoying granule was applied. It has been reported that firmicute flora is the unique flora of obesity [12]. Hashimoto's thyroiditis generally changes from the hyperthyroidism stage to the hypothyroidism stage, during which there is often a trend of weight loss, and gradually entering the hypothyroidism stage, the metabolism of the human body slows down, which is easy to lead to obesity. Whether the results of this experiment are related to obesity needs further verification. An experiment conducted by Founder found that firmicufirma increased in depressed patients compared with healthy patients [13–16]. While Ganyuqi and spleen deficiency are caused by liver loss and dreariness, liver qi stagnation, and cross and reverse invasion of the spleen. It leads to spleen deficiency, often depressed, uncomfortable, not thinking about eating and other symptoms, which are consistent with depression, poor mood, loss of appetite and other symptoms. At class level, the number of clostridium in the model group was higher than that in the normal group, while the number of clostridium in the traditional Chinese medicine group was lower. Studies have shown that the colonization of clostridium intestinalis can effectively induce the production of IL-17 and IL-22 by CD4 helper T cells (namely Th17 cells) in the lamina propria of the intestinal mucosa, and the more Th17 cells detected in the lamina propria of the intestinal mucosa, the more clostridium colonized in the intestinal mucosa [17–20]. However, the intestinal tract with fewer Th17 cells in the lamina propria lacks clostridium colonization. Therefore, it can be speculated that Clostridium is a major immune response molecule, and its colonization promotes the production of serum amyloidA (SAA) in the terminal ileum. SAA activates the 1amina propria dendriiccells (LPDCs) of the intestinal epithelial mucosa, thereby promoting the differentiation of Th17 cells [21–23]. Research literature suggests that Th17 is involved in cellular and autoimmune thyroid diseases in the form of the IL-23/IL-17 inflammatory axis. Il-17a and I-17F produced by Th17 can mobilize, mobilize and activate neutrophils, mediating the occurrence of early inflammatory response. And IL-22 production could induce the production of antimicrobial peptides by intestinal epithelial cells. These protective factors are generated due to the colonization of Clostridium to protect the host from pathogenic microorganisms. The higher the colonization density of Clostridium is, the higher the concentration of IL-17 and IL-22 lies in its colonization site. Therefore, pathogenic microorganisms were greatly reduced in the vicinity of Clostridium colonization. However, high concentrations of cytokines can also destroy the immune homeostasis of sensitive hosts, leading to the attack on their own antigens. This will mediate the formation of autoimmune diseases. At the genus level, prevotella increased in the model group compared with the normal group, while prevotella decreased after the adjustment of the traditional Chinese medicine group. Studies have shown that the implantation of Prevotella into mice can promote the production of Th17 cells [24, 25]. Some studies have confirmed that Th17 cells are involved in the occurrence and development of Hashimoto's thyroiditis, and the elevated level of Th17 cells is positively correlated with thyroid autoimmune injury [26, 27]. However, Zhao et al. [28] conducted a study in which prevotella was reduced in patients with normal thyroid function and elevated TGAb and TPOAb. As there are several types of Hashimoto's disease with normal, overactive, and decreased thyroid function, the relationship between the difference in results and thyroid function needs to be further verified.

## 3. Animal Data

Forty-eight SPF female rats were selected as subjects, and 12 rats were randomly selected as the normal control group. The remaining rats were treated with drug intervention, restraint, overwork, and diet restriction to establish the Hashimoto rat model of liver depression and spleen deficiency. After successful modeling, the rats were randomly divided into three groups: the model group, the TCM group, and the Jinshuibao group, with 12 rats in each group. The body weight of 48 SD rats was (180–220) g, with an average of (200.00 ± 20.00) g. Animal Qualification Certificate No. SCXX-2005-0001. All the selected animals were purchased from Liaoning Growth Biotechnology Co., Ltd., and the purchased rats were placed in the animal room of Liaoning University of Traditional Chinese Medicine for 7-d adaptive feedings. The rats were fed with alternating light for 12 h.

### 3.1. Drug Reagents and Instruments

The medicine Ruanjian Xiaoying granule is made by Jiangyin Tianjiang Pharmaceutical Limited Company, and the main drug components include white peony root, angelica, buchaihu, atractylodes, poria cocos, and seaweed. Reagents include anhydrous sodium iodide (Tianjin Kemiou Chemical Reagent Co., Ltd., Batch No. Q/12HB 3847-2018), thyroglobulin (70 mg/bottle, purchased from Sigma Company in the United States, provided by Anhui Cool Bioengineering Co., Ltd.), incomplete adjuvant of Fredrin, complete adjuvant of Fredrin, (10 ml/bottle, Sigma Company in the United States, provided by Anhui Cool Bioengineering Co., Ltd.). Electronic balance, bought from Shanghai, model JH1002; Axy Prep DNA Gel Recovery Kit, purchased from AXYGEN; Quantiflourtm-st Blue Fluorescent Quantitative System, purchased from Promega, Inc.

### 3.2. Preparation Method of Primary Immunoreagents

Thyroglobulin was dissolved in phosphate buffer to make an antigen solution with a concentration of 1 mg/ml. Complete fredrin adjuvant was added in equal volume to achieve full emulsification. The preparation method of booster immunoreagent was the same as that of primary immunoreagent, except that complete Freund's adjuvant was replaced by incomplete Freund's adjuvant.

## 4. The Proposed Method

### 4.1. Modeling Method of Hashimoto's Thyroiditis Model

The model of Hashimoto's thyroiditis was induced by high iodine water combined with complete Freund's adjuvant and incomplete F reund's adjuvant immunoreagent. The specific methods were as follows: After one week of adaptive feeding, the blank group drank distilled water, and the other blank group drank high iodine water (concentration of 0.64 g/L). From the fourth week, except the blank group, all rats were injected subcutaneously with 0.2 ml of primary immune reagent containing complete Fredrin's adjuvant antigen twice a week. From the 5th to 8th week, 0.2 ml of immunobooster reagent with incomplete Freund's adjuvant antigen was injected once a week.

### 4.2. Modeling Method of the Liver Depression and Spleen Deficiency Model

TCM syndrome type building method, using the bound stress, fatigue, and diet not festival made change model compound mode [29]. The fifth week, all except the blank group rats in a cylinder are bound to limit activities, 1 hour/day, put in the rat swimming pool until the rat physical drains out, 1 time/day, and the blank group daily to a normal rat feed. The other rats were fed every other day for 4 weeks.

### 4.3. Treatment Methods of Rats

All the animals were fed adaptively for 7 days, and the rats were routinely divided into groups. At week 2, the normal group was given distilled water intervention, while the model group, TCM group, and Jinshuibao group were given high iodine water. From the 4th week, each group (except the normal group) was immunized by multi-point injection under foot, and from the 5th week to the 8th week, a booster immunizer was injected once a week. From the fifth week, the blank group was fed with feed every day, and the other three groups were placed in the restraint tube for one hour to restrict free movement, then placed in the bucket for swimming until exhaustion, and fed with feed the next day.

### 4.4. Drug Administration Method in Rats

The normal group and model group were given 2 mL distilled water intragastric administration, twice a day. Traditional Chinese medicine group was given by Ruanjian Xiaoying granule, twice a day, the dose was 12.96 g/kg/day. In jinshuibao group, Jinshuibao capsule was dissolved in water and gavaged twice a day according to the crude drug dose of 0.45 g/kg/day for 12 weeks.

### 4.5. Determination Method of Intestinal Flora

Twelve weeks after the intervention, 9 rats in the normal group, the model group, the Ruanjian Xiaoying group, and the Jinshuibao group were removed, placed in sterile vessels, and collected by the tail lifting reflex method, with 3 rats in each group. Total genomic DNA was extracted by the CTAB/SDS method and detected by 1% agarose gel electrophoresis. The DNA was diluted to 1 ng/*μ*L using diluent. PCR amplification was performed on extracted genomic DNA. PCR products were monitored by 2% agarose gel electrophoresis, and PCR products were recovered by the AxyPreDNA gel recovery kit. A Quantiflourtm-st blue fluorescence quantitative system was used to recover the quantitative PCR amplification products. Using 16S DNA amplicon sequencing, the species composition of samples can be revealed by splicing and filtering reads, clustering of Operational Taxonomic Units (OTUs), species annotation and abundance analysis, and furthermore, differences between samples can be mined to screen for differential flora.

### 4.6. OTU Classification and Classification Status Identification

Using 97% sequence similarity as the OTU (Operational Taxonomic Unit) classification threshold, which roughly corresponds to sequence differences at the species level in taxonomy, OTU whose abundance value was less than 0.001% (1/100, 000) of the total sequencing amount of all samples were removed, and the abundance matrix of OTU in each sample was constructed according to the number of sequences contained in each sample. According to OTU classification and classification status identification results, the specific composition of each sample in phylum, class, order, family, and genus was obtained.

### 4.7. Data Statistical Methods

The SPSS 22.0 software was used for statistical analysis and GraphPad Prism 5.0 was used for plotting. The measurement data of normal distribution were expressed as ($\bar{x}$ ± *s*), and the independent sample *T*-test was used for comparison between the two groups. Non-normally distributed data were expressed as the median (interquartile spacing), and comparisons between the two groups were performed using the Mann-Whitney rank-sum test. *P* < 0.05 indicated that the difference was statistically significant.

## 5. Experimental Data

### 5.1. Modeling of Mice

There were 9 rats in the normal group, the model group, the Ruanjian Xiaoying group, and the Jinshuibao group, respectively. Compared with the normal group, the total movement distance and the number of holes in the central region of the model group were significantly reduced, with statistical significance (See Table 1). The fecal water content of rats in the model group increased, which was statistically significant (see Table 2), proving that the model of liver depression and spleen deficiency was successfully replicated. TGAb and TPOAb increased significantly in the model group, and the differences were statistically significant, indicating that the Hashimoto's thyroiditis model was successfully replicated, as shown in Table 3. At the same time, the model group showed symptoms of liver depression and spleen deficiency, dark, coarse, and dull hair, decreased activity, clustering and arching back, decreased eating, and even occasionally loose stools.

### 5.2. Conditions of Rats in Each Group after Treatment

After treatment, compared with model group, TGAb and TPOAb of the TCM group and Jinshuibao group decreased significantly, and the difference was statistically significant, indicating that both Ruanjian Xiaoying granule and Jinshuibao had certain therapeutic effects. At the same time, compared with model group, the hair color of the soft and firm eliminating gall group was shinier, activity increased, eating was acceptable, and there were no loose stools. The hair color of the Jinshuibao group was slightly shiny, and the symptoms of eating and loose stools were improved compared with the model group, as shown in Table 4. It should be noted that the comparison was conducted between the postmold making model group and the normal group and  ^*∗*^*P* < 0.05. The Ruanjian gall group was compared with the model group and ^#^*P* < 0.05. After treatment, the Campbell group was compared to the model group and ^##^*P* < 0.05.

### 5.3. A Venn Plot Based on the OTU Distribution

Among them, by using the R software, the number of OTUs in 4 groups was calculated based on the obtained OTUs abundance matrix. Then, the number of common and unique OTU occupied in 4 groups can be visually presented in by drawing the Venn plot of OTUs. As shown in Figure 1, 44 OTU were unique to each group, 245 OTU unique to group B, 45 OTU unique to group C, and 124 OYU unique to group D, with 1033 OTU overlapping each other, where A, B, C, and D represent the normal group, model group, Chinese medicine group, and Jinshuibao group, respectively.

### 5.4. Composition Diagram of Community Structure

At the phylum level, firmicutes increased and proteobacteria decreased in the model group compared with the normal group. Firmicutes were reduced in the Chinese medicine group after the treatment with Ruanjian Xiaoying granules. Proteobacteria increased. However, the Jinshuibao group could make firmicutes and proteobacteria closer to the normal group, as shown in Figure 2.

According to the obtained community structure composition diagram of the class, the number of Clostridium in the model group was significantly higher than that in the normal group. Besides, the number of Clostridium in the traditional Chinese medicine group was significantly lower than that in the model group. While the number of Clostridium in the Jinshuibao group was not significantly decreased, as shown in Figure 3.

At the genus level, the number of Eschia and flavor-like bacteria in the model group was significantly reduced compared with the normal group, while the number of Prevotella was increased compared with the normal group. The Chinese medicine group had a regulatory effect on the above three bacteria genera closer to the normal group, while the Jinshuibao group had no such regulatory effect, as shown in Figure 4.

## 6. Conclusions

In this study, experiments were conducted on the intestinal flora of rats with liver depression and spleen deficiency. Intestinal flora is an important part of gastrointestinal function, which is involved in the whole process of physiology, biochemistry, pathology, and pharmacology. Experimental results show the application of Ruanjian Xiaoying granules in Hashimoto rats with liver depression and spleen deficiency can improve serum TGAb and TPOAb levels, regulate thyroid function and promote the recovery of organism flora levels, providing ideas for the treatment of Hashimoto thyroiditis.

## Figures and Tables

**Figure 1:** Venn diagram of OTU distribution.

**Figure 2:** Composition of fecal microflora in each group of mice.

**Figure 3:** Composition diagram of fecal microflora in each group.

**Figure 4:** Composition diagram of fecal microorganisms in each group.

**Table 1:** Comparison of open field experiment between the two groups of rats ($\bar{x}$ ± *s*).

The truancy experiment Total movement distance of 5 min movement (cm)	*n*	Normal group		Model set	
		Before mold making	After mold making	Before mold making	After mold making
Total movement distance in the central area (cm)	9	2578.9 ± 225.0	1933.9 ± 126.3	2774.9 ± 128.1	1163.9 ± 107.6 ^*∗*^
Number of grids in central area (times)	9	74.3 ± 7.5	87.4 ± 6.3	71.1 ± 5.9	81.7 ± 6.7
Stay time in the central zone (s)	9	101.9 ± 6.5	78.7 ± 5.6	105.3 ± 8.0	38.7 ± 4.6 ^*∗*^
The truancy experiment	9	6.7 ± 1.1	8.3 ± 1.1	6.4 ± 0.9	9.1 ± 1.3

**Table 2:** Comparison of water content in feces between the two group ($\bar{x}\pm s$).

Group	*n*	Before mold making	After mold making
Normal group	9	29.6 ± 4.9	28.9 ± 5.3
Model set	9	28.9 ± 4.4	39.8 ± 4.6 ^*∗*^

**Table 3:** Comparison of TGAb and TPOAb in rats ($\bar{x}\pm s$).

Group	*n*	Time	TGAb (IU·ml^−1^)	TPOAb (IU·ml^−1^)
Normal group	9	After mold making	96.8 ± 12.8	9.9 ± 1.5
Model set	9	After mold making	177.0 ± 17.2 ^*∗*^	17.7 ± 1.6 ^*∗*^

**Table 4:** Serum levels of TGAb and TPOAb in rats from each group after treatment ($\bar{x}\pm s$).

Group	*n*	Time	TGAb (ng/ml)	TPOAb (pg/ml)
Normal group	9	Posttreatment	98.3 ± 11.7	9.68 ± 1.5
Model set	9	Posttreatment	184.5 ± 27.0 ^*∗*^	17.5 ± 2.9 ^*∗*^
Ruanjian elimination gall group	9	Posttreatment	130.0 ± 7.7^#^	12.7 ± 1.2^#^
Jinshuibao group	9	Posttreatment	130.9 ± 12.4^##^	13.2 ± 1.5^##^

## Data Availability

The simulation experiment data used to support the findings of this study are available from the corresponding author upon request.
